# The Prepless Approach for Cantilever Resin-Bonded Bridge Using Computer-Aided Design and Manufacturing Technology for the Minimally Invasive Replacement of a Maxillary Central Incisor: A Case Report of a Rare Procedure

**DOI:** 10.7759/cureus.91872

**Published:** 2025-09-08

**Authors:** Hariri Ismail, Dabla Fahd, Zeyneb El Maddah El Idrissi, Amal El Yamani

**Affiliations:** 1 Prosthodontics Department, Faculty of Dental Medicine, Mohammed V University, Rabat, MAR

**Keywords:** case report, computer aided design, computer aided manufacturing, minimally invasive dentistry, resin bonded bridge

## Abstract

Replacing a maxillary central incisor in young patients presents both aesthetic and functional challenges, particularly when implant therapy is contraindicated due to ongoing post-pubertal craniofacial growth. This case report describes the use of a prepless cantilever resin-bonded fixed dental prosthesis fabricated from lithium disilicate using a Computer-Aided Design and Computer-Aided Manufacturing (CAD/CAM) workflow to restore a maxillary central incisor in a 20-year-old female patient. The treatment involved selective removal of aprismatic enamel without conventional tooth preparation, promoting dental tissue preservation and adhesion. A silicone repositioning index ensured accurate clinical placement of the bridge. At 20 months, the restoration demonstrated excellent aesthetic, biological, and functional integration. This technique represents a reliable, conservative, and aesthetic alternative to implants in carefully selected young patients.

## Introduction

The loss of a maxillary central incisor can be particularly distressing for patients, both psychologically and socially, as it significantly affects well-being, mastication, and even phonation. To address the absence of this anterior tooth, a range of therapeutic options are available: removable prostheses, fixed partial dentures, and dental implants. Among these, the cantilever resin-bonded bridge with a single wing, first proposed by Matthias Kern [1], presents a viable and conservative alternative to conventional fixed partial dentures, which require substantial preparation of adjacent teeth. Numerous studies, including that of Mine et al., have reported a 100% survival rate over a 10-year follow-up period, thereby confirming the long-term success of this treatment approach [2]. This technique aligns closely with the principles of minimally invasive dentistry, especially in young patients who may exhibit residual post-pubertal craniofacial growth that could compromise the long-term success of implant therapy. The main complications reported include the infraocclusion positioning of dental implants in the maxillary arch and the rotation of dental implants in the mandibular arch [3].

Several studies have described the standardized minimal preparation protocol for the abutment tooth, as advocated by Professor Matthias Kern [1], before impression taking. In this case report, we highlight an original conservative strategy: a prepless approach, in which only the aprismatic enamel is gently removed, without any conventional tooth preparation, for the replacement of the right maxillary central incisor using a cantilever resin-bonded bridge. The restoration was fabricated from lithium disilicate glass-ceramic using a Computer-Aided Design and Computer-Aided Manufacturing (CAD/CAM) workflow, in a healthy 20-year-old female patient with no signs of parafunctional habits. This report demonstrates the feasibility and favorable short- to mid-term clinical outcome (20 months) of a prepless CAD/CAM cantilever resin-bonded bridge used to replace a maxillary central incisor in a young adult patient.

## Case presentation

A 20-year-old female patient presented to the department of fixed prosthodontics in January 2024 seeking urgent prosthetic rehabilitation following the loss of her maxillary right central incisor. The patient explicitly refused any preparation of adjacent teeth. Her chief concern was aesthetic, as the missing tooth had a significant psychological impact. She was in good general health with no identified parafunctional habits. The tooth had been rendered unrestorable due to a road traffic accident and subsequently extracted. Given the pressure of intensive academic studies, she requested a rapid fixed solution.

Before the prosthodontic consultation, the patient had undergone orthodontic treatment to reorganize the dental arch and ensure a stable occlusion. This included a palatal arch appliance with a resin tooth replacing the missing incisor. Subsequently, she wore a thermoplastic retainer with a provisional tooth, which she found uncomfortable, prompting her to seek a fixed prosthetic alternative.

Clinical and radiographic findings

Extraorally, the patient presented with a harmonious facial appearance and a normal vertical dimension of occlusion (VDO), with no signs of temporomandibular disorders. Clinical examination intraorally revealed the absence of the right central incisor, with slight ridge resorption. Oral hygiene was satisfactory, and the gingiva appeared pink and healthy. The adjacent left central incisor, designated as the abutment tooth, was caries-free, properly aligned, and presented an adequate enamel surface suitable for optimal bonding (Figure 1A). It exhibited a healthy periodontium, with 5 mm of keratinized gingiva. No periodontal pockets were detected (probing depth ≤3 mm) around this tooth, and it exhibited sufficient alveolar bone support. No mobility (Miller Class 0) was observed; no gingival recession was detected, and no loss of attachment was determined.

**Figure 1:** A: Initial situation - the right central incisor was missing with slight ridge resorption. The adjacent left central incisor, selected as the abutment, was caries-free, in proper alignment, with a healthy periodontium. Gingival tissues appeared healthy. B: left view showing stable occlusion. C: right view showing stable occlusion

The lateral incisor was excluded as a potential abutment due to its smaller bonding surface. Occlusal evaluation confirmed a harmonious distribution of occlusal contacts on both the left and right sides, indicating a stable maximum intercuspation, with the absence of any dental lesions such as abfractions or other defects (Figures 1B, 1C). Radiographic examination revealed no signs of endodontic or periodontal pathology, with no bone defects observed. Taken together, these clinical and radiographic findings confirmed that the left central incisor was the most suitable abutment for the prepless cantilever resin-bonded bridge.

Diagnosis and therapeutic decision

A primary impression was taken to analyze the edentulous space, followed by a diagnostic wax-up of the right central maxillary incisor to assess the available space and global aesthetic result. The chosen treatment plan involved the fabrication of a cantilever resin-bonded fixed dental prosthesis in lithium disilicate, using a prepless approach and relying solely on the left central incisor as the abutment, with fabrication via CAD/CAM technology. This plan addressed the patient's urgent demand and aesthetic goals while preserving the structural integrity of the left central incisor. A dental implant to replace the right maxillary central incisor was excluded due to time constraints and the risk of residual post-pubertal growth potentially resulting in infraocclusion of the implant-supported prosthesis. The treatment plan was thoroughly explained to the patient, and informed consent was obtained.

Removal of aprismatic enamel and impression taking

The initial clinical step involved selective removal of aprismatic enamel, known to hinder optimal adhesion, using a fine-grit diamond bur, followed by shade selection (Figure 2). After verification, a single-step impression was performed using polyvinyl siloxane as the impression material to produce the working model (Figure 3).

**Figure 2:** Removal of aprismatic enamel using a fine-grit diamond bur (prepless approach) No preparation design was performed; only superficial enamel removal was carried out

**Figure 3:** One-step impression technique using polyvinyl siloxane as the impression material

Digital workflow steps and fabrication of a silicone repositioning index

To optimize visualization and prosthesis design, a digital workflow (CAD/CAM) was employed. Maxillary and mandibular models, along with their occlusion, were scanned. The first design step was to define the limits of the wing extension over the palatal surface of the left maxillary central incisor (Figure 4A), followed by three-dimensional design of the pontic to mirror the contralateral incisor, and finally the connector (Figures 4B, 4C). To prevent premature fracture and to comply with the mechanical requirements of lithium disilicate glass-ceramics, the connector area was defined with a 12 mm² surface. Milling was carried out using a five-axis milling machine.

**Figure 4:** A: Delineation of the limits of the future wing. B: Digital design of the pontic and connector in the palatal view. C: Digital design of the pontic in the buccal view

Due to the absence of mechanical retention and the risk of misplacement, a silicone repositioning index was fabricated in the laboratory to ensure accurate bridge placement; a midline reference mark was used to minimize the risk of mispositioning (Figure 5A); the index was trimmed to ensure accurate placement (Figure 5B), facilitate both the supporting of the prosthetic reconstruction and the removal of excess cement during bonding (Figure 5C).

**Figure 5:** A: Vertical line traced within the index served as a reference mark for the midline, ensuring correct alignment and minimizing the risk of mispositioning. B: The index was carefully trimmed to optimize handling, enable precise placement, and allow efficient removal of excess cement during bonding. C: Prosthetic restoration supported by the repositioning index

Final try-in and bonding protocol

Two days later, the restoration was delivered, and a clinical trial verified both marginal adaptation and aesthetic integration. Following validation, the bonding protocol was carried out as follows: the intaglio surface of the prosthesis was etched with 5% hydrofluoric acid for 30 seconds (Figure 6A), in accordance with the guidelines for lithium disilicate bonding. A characteristic chalky appearance was observed (Figure 6B). To remove any etching residue that could impair adhesion, the intaglio surface was further conditioned with 37% phosphoric acid for 120 seconds (Figure 6C). The intaglio surface after this procedure was clean and ready for bonding (Figure 6D). This step was followed by the application and two-minute evaporation of a silane coupling agent (Figure 6E).

**Figure 6:** A: Etching of the ceramic surface with 5% hydrofluoric acid for 30 seconds to create micro-roughness, allowing infiltration of the silane coupling agent. B: Chalky white appearance observed after acid etching, rinsing, and drying corresponds to hydrofluoric acid etching residues, which, if not removed, may reduce adhesion values and compromise bonding. C: Application of 37% phosphoric acid to neutralize the chalky white appearance. D: Clean prosthetic intaglio surface prepared and optimized for bonding, as indicated by the disappearance of the chalky white appearance. E: Application of silane coupling agent on the intaglio surface to improve chemical bonding between the ceramic and the resin cement

The abutment tooth was etched with 37% phosphoric acid for 30 seconds (Figure 7A), as the bonding surface was entirely within enamel. It was then rinsed, air-dried (Figure 7B), and coated with adhesive (Figure 7C), which was light-cured for 20 seconds (Figure 7D).

**Figure 7:** A: Etching with 37% phosphoric acid. B: Rinsing and drying. C: Application of adhesive. D: Light curing

The prosthesis was bonded using a dual-cure adhesive resin cement. The silicone index facilitated precise positioning (Figure 8A). Excess cement was removed, and each surface was light-cured for 20 seconds (Figure 8B) (repeated three times). The entire bonding procedure was performed under rubber dam isolation to ensure optimal moisture control.

**Figure 8:** A: Placement of the cantilever resin-bonded bridge with resin cement applied to the intaglio surface of the retainer wing, using the repositioning index. B: Light-curing after placement of the cantilever resin-bonded bridge to ensure proper polymerization of the resin cement

Outcome and follow-up

Following rubber dam removal, the outcome was evaluated. Intraorally, the restoration demonstrated harmonious adaptation to the adjacent teeth (Figure 9A), while extraorally it exhibited an aesthetically pleasing integration within the smile, with appropriate color match and natural appearance (Figure 9B). Occlusal adjustments were performed after bonding.

**Figure 9:** A: Intraoral examination immediately after bonding revealed a harmonious adaptation of the restoration to the adjacent teeth. B: The extraoral view demonstrated an aesthetically pleasing integration within the smile, characterized by appropriate color matching and a natural appearance

At the 20-month follow-up, the prosthesis demonstrated excellent aesthetic, functional, and biological integration (Figures 10A, 10B). The patient expressed high satisfaction with the aesthetic result and reported a renewed sense of confidence in her smile. (Figure 10C). She presented with normal functional mandibular movements and no signs of temporomandibular joint disorders.

**Figure 10:** A: Frontal view demonstrating excellent biological and aesthetic integration at the 20-month follow-up. B: Lateral view illustrating the natural appearance of the prosthetic reconstruction. C: The patient’s harmonious and confident smile

Oral hygiene instructions, including the use of interdental brushes and dental floss, were explained at the beginning of treatment and maintained consistently, resulting in effective plaque control. The periodontal tissues remained healthy, with 5 mm of keratinized gingiva at the abutment site, no probing depths beyond 3 mm, and no signs of gingival recession, attachment loss, or abutment mobility. The preparation was limited to an aprismatic enamel, ensuring a stable adhesion. The wing thickness (0.8 mm) and connector dimensions (12 mm², 4 mm height × 3 mm width) remained intact without signs of stress or fracture. Occlusion was stable, with the wing margins positioned outside functional contacts and no pontic involvement in dynamic occlusion. Both the ceramic and abutment maintained structural integrity, and no fractures or debonding were observed. Aesthetically, the restoration demonstrated natural color and contour harmony, leading to satisfactory integration. Overall, at the 20-month follow-up, functional, aesthetic, and biological outcomes were stable.

## Discussion

The resin-bonded bridge, first introduced by Rochette in 1972 [4], was initially designed with two perforated wings without any tooth preparation. However, this type of restoration exhibited a high failure rate [5], which led to its abandonment for long-term rehabilitation. Advances in the understanding of the biomechanics of such bonded bridges, particularly the mechanisms of debonding, have highlighted the issue of differential mobility between abutment teeth, often leading to debonding of the wing attached to the weaker tooth [6]. These observations prompted Kern and his collaborators to develop the cantilever approach. According to a study by Kern and Sasse, this technique achieved a survival rate of 94.4% over 10 years when fabricated in zirconia [7], making it a reliable long-term solution. Although initially indicated for the replacement of maxillary lateral incisors [8], this technique has since been extended to the replacement of central incisors and even first premolars [9].

The materials used are typically zirconia or lithium disilicate. While a standardized preparation design as recommended by Mathias Kern is generally employed to ensure optimal stability for the resin-bonded cantilever bridge [1], we adopted a "prepless" approach, limited to the removal of aprismatic enamel. This strategy aims to maximize residual enamel conservation, thus ensuring optimal adhesion; as is known, aprismatic enamel constitutes a barrier to acid etching, thereby complicating adhesive protocols and posing a challenge for achieving predictable bonding effectiveness [10]. This method also aligns with the principles of minimally invasive dentistry. In the study by Sailer et al., 40 patients received 49 cantilever single-retainer glass-ceramic replacing central and lateral incisors, premolars, and two molars. For the anterior abutments, no preparation design was performed. No fractures or removals due to technical or biological complications occurred (95% CI: 0.00-10.00%), resulting in a five-year survival rate of 100% (95% CI: 90-100%) [11].

Sillam et al. demonstrated that a localized preparation of a 12 mm² box provides better shear resistance than an extended preparation of the dental surface [12]. Recently, an article by Mainjot described 16 zirconia cantilever resin-bonded bridges placed without any preparation design in 11 patients. The survival rate was 100% after a mean follow-up of 3.0 ± 2.6 years (range: one month-9.5 years) [13]. The only difference compared to our case is the use of zirconia instead of glass-ceramic. Together with the findings of Sailer et al. [11], these results align with the outcome of our clinical case report and support the reliability of cantilever resin-bonded bridges without a preparation design. 

Compared with dental implants, cantilever resin-bonded bridges are less invasive, more cost-effective, and avoid implant-related complications such as peri-implantitis. They are particularly indicated in cases of insufficient bone height or thickness, unfavorably angulated roots, in young patients, or in individuals with medical contraindications to implant surgery [13]. Also in comparison with conventional fixed partial dentures, cantilever resin-bonded bridges allow for superior tissue preservation [11], thereby avoiding postoperative pulp sensitivity or pain suggestive of pulpal pathology. Contemporary evidence indicates that the clinical performance of cantilever resin-bonded bridges is now comparable to that of conventional fixed partial dentures and implant-supported crowns, with a five-year success rate of 88% for metal cantilever resin-bonded bridges and 84% for non-metal cantilever resin-bonded bridges. Consequently, the cantilever resin-bonded bridge is increasingly recognized as a reliable alternative to conventional fixed partial dentures and implant-supported crowns. This trend is particularly relevant in the anterior zone, where aesthetic demands are greater, the risk of infraposition with implants is more problematic, and occlusal forces are comparatively lower than in the posterior region [13]

The integration of CAD/CAM technology has enabled enhanced three-dimensional morphological control, particularly regarding connector thickness, thereby reducing the risk of premature fracture [14]. A comparative study in 2014 revealed that restorations fabricated via digital workflow demonstrated better marginal accuracy (48 ± 25 µm) than those produced using conventional techniques (74 ± 47 µm) [15]. Moreover, a finite element analysis conducted by Keulemans et al. showed that stress concentration was greatest at the connector, underscoring the critical importance of its design [16]. The use of a silicone repositioning index improved placement precision, avoiding malpositioning that could compromise occlusion [17].

A fundamental criterion for success lies in the stability of the occlusion. The margins of the wing must be located outside the zones of occlusal contact [1]. Particular attention should be paid to parafunctional habits (pen chewing, onychophagia). Kern emphasizes that anterior guidance should not be delegated to the pontic in lateral or protrusive movements; this function must remain with the abutment tooth. Failure to respect this principle could lead to abutment tooth rotation, loss of proximal contact, and compromised prosthetic stability. To prevent complications arising from nocturnal parafunctions, the author recommends the use of a thermoformed night guard (2 mm thickness), adjusted to the patient's occlusion [18]. Bonding is performed using an adhesive resin composite containing MDP (10-methacryloyloxydecyl dihydrogen phosphate) monomer for zirconia, whereas a dual-cure adhesive resin cement is used for lithium disilicate [19]. In our case, we followed recommendations in the recent literature, particularly the use of a second phosphoric acid etching step after the initial hydrofluoric acid etching, to optimize adhesion [20].

Despite its many advantages, the cantilever resin-bonded bridge has some limitations. It requires strict case selection (absence of parafunctions, sufficient enamel, inadequate occlusal space less than 0.7 mm) [13], a rigorous bonding protocol, and impeccable oral hygiene. In case of debonding, repair can be complex and necessitates close follow-up. Additionally, access to CAD/CAM technology may be limited, restricting its use in daily practice. Finally, the follow-up period in our case is currently limited to 20 months, calling for longer-term evaluation. Few studies have investigated the “prepless” approach, warranting further research to validate its long-term clinical performance.

## Conclusions

The ceramic cantilever resin-bonded bridge, when combined with a prepless approach and CAD/CAM technology, represents a promising, aesthetic, and minimally invasive treatment option for replacing a maxillary central incisor, particularly in young patients who are not suitable candidates for implant therapy. The absence of conventional tooth preparation preserves the abutment enamel, which is fundamental for optimal bonding, while a meticulous adhesive protocol ensures favorable short- to mid-term performance, as seen in our case. The 20-month follow-up findings support its clinical potential. Although these observations are based on a single case, the outcome aligns with longer-term results reported in the literature, suggesting the reliability of this therapeutic approach. Nevertheless, further clinical investigations are necessary to confirm its long-term applicability.
